The article "Ras-ERK1/2 signaling contributes to the development of colorectal cancer via regulating H3K9ac" was retracted in 2021. Reasons: manipulated images; duplicated images; signs of a paper mill; unreliable data.

# Ras-ERK1/2 signaling contributes to the development of colorectal cancer via regulating H3K9ac

**DOI:** 10.1186/s12885-018-5199-3

**Published:** 2018-12-22

**Authors:** Peng Tian, Yanfei Zhu, Chao Zhang, Xinyu Guo, Peng Zhang, Huanzhou Xue

**Affiliations:** 1 Department of Gastrointestinal Surgery, Zhengzhou University People’s Hospital (Henan Provincial People’s Hospital), Zhengzhou, 450003 China; 2 Department of General Surgery, Wuxi People’s Hospital of Nanjing Medical University, Wuxi, 214023 China; 3 Department of General Surgery, Zhengzhou University People’s Hospital (Henan Provincial People’s Hospital), No.7, Weiwu Road, Zhengzhou, 450003 Henan China

**Keywords:** Ras, ERK1/2, H3K9ac, HDAC2, PCAF, Colorectal cancer

## Abstract

**Backgrounds/aims:**

Ras is a control switch of ERK1/2 pathway, and hyperactivation of Ras-ERK1/2 signaling appears frequently in human cancers. However, the molecular regulation following by Ras-ERK1/2 activation is still unclear. This work aimed to reveal whether Ras-ERK1/2 promoted the development of colorectal cancer via regulating H3K9ac.

**Methods:**

A vector for expression of *K-Ras* mutated at G12 V and T35S was transfected into SW48 cells, and the acetylation of H3K9 was measured by Western blot analysis. MTT assay, colony formation assay, transwell assay, chromatin immunoprecipitation and RT-qPCR were performed to detect whether H3K9ac was contributed to K-Ras-mediated cell growth and migration. Furthermore, whether HDAC2 and PCAF involved in modification of H3K9ac following Ras-ERK1/2 activation were studied.

**Results:**

*K-Ras* mutated at G12 V and T35S induced a significant activation of ERK1/2 signaling and a significant down-regulation of H3K9ac. Recovering H3K9 acetylation by using a mimicked H3K9ac expression vector attenuated the promoting effects of Ras-ERK1/2 on tumor cells growth and migration. Besides, H3K9ac can be deacetylated by HDAC2 and MDM2-depedent degradation of PCAF.

**Conclusion:**

H3K9ac was a specific target for Ras-ERK1/2 signaling pathway. H3K9 acetylation can be modulated by HDAC2 and MDM2-depedent degradation of PCAF. The revealed regulation provides a better understanding of Ras-ERK1/2 signaling in tumorigenesis.

## Background

Ras is a small GTPase. It has been considered as a control switch of ERK/MAPK pathway, and both of Ras and its downstream signaling effector ERK/MAPK can modulate the activation of PI3K, mTOR and AMPK pathways [1]. Because of that, Ras plays a pivotal role in regulating multiple cellular responses, such as proliferation, differentiation, apoptosis, senescence, metabolism [2], and even cancer initiation and progression [3]. Ras protein is encoded by three ubiquitously expressed genes: *H-Ras*, *K-Ras* and *N-Ras*, among which *K-Ras* shows significant carcinogenesis when mutated at codon 12 [4]. In this process, Glycine (G) in position of codon 12 is replaced by Cysteine (C), Asparticacid (D), Serine (S), Arginine (R) or Valine (V). Of note, G12 V together with T35S and V45E are most widely studied mutation sites of *Ras*. As reported by Catalogue Of Somatic Mutations In Cancer (COSMIC), the incidence of *K-Ras* point mutation in human cancers is approximately 30%, with pancreatic cancer accounting for 90%, colorectal cancer for 45%, and non-small cell lung cancer for 35% (https://cancer.sanger.ac.uk/cosmic).

The article "Ras-ERK1/2 signaling contributes to the development of colorectal cancer via regulating H3K9ac" was retracted in 2021. Reasons: manipulated images; duplicated images; signs of a paper mill; unreliable data.

In eukaryotic cells, nucleosomes are composed of two each of histones H2A, H2B, H3 and H4. Recently, histone modification has been widely explored since its important role in regulating tumorigenesis [5]. In the field of histone modification, histone acetylases (HATs) and histone deacetylases (HDACs) are involved in alteration of the chromatin structure, of which modulating gene transcription. HDAC2, one type of HDACs, locates in nucleus and can function alone. It modulates gene expression by deacetylating the N-terminal tails of the core histones, resulting in the tightening of the chromatin, which reduces its accessibility for the transcriptional machinery [6]. Recent years, acetylation of histone H3 has become a hot topic in epigenetic regulation [7]. One of the widely studied acetylation site of histone H3 tails is histone H3 lysine 9 (H3K9), produces the acetylated lysine 9 of histone H3 (H3K9ac). H3K9ac is also essentially related to transcriptional activation in human cells, and its hypoactivation is closely associated with the occurrence and development of multiple types of cancer [7, 8]. More interestingly, H3K9ac can be specifically modulated by HDAC2 in oligodendrocyte [9]. However, the role of H3K9ac in colorectal cancer has not been well-studied yet.

Previous studies have suggested that deregulation of Ras signaling led to aberrant histone modification, resulting in cancer development. For instance, Ras-PI3K-AKT pathway regulated histone H3 acetylation at lysine 56 (H3K56ac) via the MDM2-dependent degradation, and thus regulating tumor cells activity [10]. Another study demonstrated that Ras signaling showed oncogenic role through regulating histone covalent modifications [11]. In this study, we established a link between Ras signaling and H3K9ac modification, aiming to reveal one of the underlying mechanisms of which *K-Ras* point mutation contributed to colorectal cancer cells growth and migration.

## Methods

### Cell culture and treatment

Human colorectal cancer cell line SW48 purchased from American Type Culture Collection (Catalogue number: CCL-231™, ATCC, Manassas, VA, USA) was cultured in Dulbecco’s Modified Eagle’s Medium (DMEM, Gibco, Grand Island, NY, USA) supplemented with 10% heat-inactivated fetal bovine serum (FBS, Gibco). The cells were maintained at 37 °C in a humidified atmosphere with 5% CO_2_.

The article "Ras-ERK1/2 signaling contributes to the development of colorectal cancer via regulating H3K9ac" was retracted in 2021. Reasons: manipulated images; duplicated images; signs of a paper mill; unreliable data.

MG132 (≥95% HPLC), an inhibitor of proteasome, was purchased from Sigma-Aldrich (St. Louis, MO, USA). SW48 cells were treated by 25 μM MG132 for 0–12 h. SCH772984, SB203580, LY294002 and SP600125, the specific inhibitors for ERK1/2, MAPK, PI3K and JNK pathways were all purchased from Selleck Chemicals (Houston, TX). These inhibitors were used with concentrations of 4 nM, 5 μM, 0.5 μM and 40 nM for treating cells for 12 h.

### Plasmid construction and cell transfection

The coding regions of human wild-type *K-Ras* and *H3* were amplified by PCR and were subcloned into pEGFP-N1 plasmid (Clontech Inc., Palo Alto, CA). The amplified *PCAF* and *HDAC2* were subcloned into pcDNA6.0/HA-tag vector (Invitrogen, Carlsbad, CA, USA). The pEGFP-K-Ras^G12V/T35S^ construct was mutated using site-directed mutagenesis. The pEGFP-H3K9Q construct was constructed using the TaKaRa MutanBEST Kit (#D401, TaKaRa, Dalian, China). Two different sequences of siRNAs specific for *HDAC2* (si-HDAC2–1 and si-HDAC2–2) were purchased from GenePharma (Shanghai, China). A non-targeting sequence was used as a negative control (si-con). MDM2-MU for expression of *MDM2*^*C464A*^ was constructed and recombination into pIB/V5-His Vector (Invitrogen).

SW48 cells were seeded in 6-well plates with a density of 1 × 10^5^ cells/well. When 50% confluence was researched, the cells were transfected with plasmids or siRNAs by using lipofectamine 3000 (Invitrogen). At 48 h of transfection, the culture medium was replaced by the complete medium to stop transfection. Transfection efficiency was confirmed by using Western blot and/or RT-qPCR.

### Cell viability

The transfected SW48 cells were collected by using trypsin (Sigma-Aldrich) and were seeded in 96-well plates with a density of 5 × 10^3^ cells/well. After 48 h of incubation at 37 °C, 20 μL of MTT solution (Sigma-Aldrich) with a final concentration of 5 mg/mL was added into each well and the plates were incubated at 37 °C for another 4 h. Then, the culture medium was removed and 100 μL dimethyl sulfoxide (DMSO, Sigma-Aldrich) was added. Following 10 min of shaking in an ELISA reader (Bio-Rad Laboratories, Hercules, CA, USA), the absorbance of each well was recorded at 570 nm.

### Transwell migrGation assay

The transfected SW48 cells were collected and seeded in the upper side of 24-well transwell chamber with 8-μm pore filters (Costar, Boston, MA). The cells were maintained at serum-free culture medium. The lower side of the chamber was filled with 600 μL complete culture medium. After 12 h of incubation at 37 °C, the cells migrated into the lower side were fixed with methanol and stained with 0.5% crystal violet (Beyotime, Shanghai, China). The absorbance of cells that had been washed with acetic acid was measured at 570 nm.

The article "Ras-ERK1/2 signaling contributes to the development of colorectal cancer via regulating H3K9ac" was retracted in 2021. Reasons: manipulated images; duplicated images; signs of a paper mill; unreliable data.

### RNA extraction and RT-qPCR

Total RNAs were extracted from the transfected cells by using the TRIzol reagent (Invitrogen). Five micrograms of total RNA was subjected to reverse transcription using the Transcriptor First Strand cDNA Synthesis Kit (Roche, Basel, Switzerland). FastStart Universal SYBR Green Master (Roche) was used in qPCR and each qPCR was carried out in triplicate for a total of 20 μL reaction mixtures on ABI PRISM 7500 Real-time PCR System (Applied Biosystems, Foster City, CA, USA). *GAPDH* served as an internal control. Data were analyzed according to the classic 2^−ΔΔCt^ method.

### Soft-agar colony formation assay

Low melting agarose (Thermo Scientific®, Rockford, IL, USA) with concentration of 0.5% was placed in 6-well plates, and the plates were incubated at 4 °C for 30 min. The transfected SW48 cells were seeded in 6-well with a density of 600 cells/well, and were cultured in DMEM containing 0.33% agarose at 37 °C for 2 weeks. The number of the colonies was counted microscopically.

### Western blot

Total protein was extracted from the transfected SW48 cells by using 1% Triton X-100 (Invitrogen) and 1 mM PMSF (pH 7.4) (Solarbio, Beijing, China) over ice for 30 min. The protein concentration was determined by BCA protein assay kit (Novagen, Madison, WI, USA). Equal amount of protein samples were subjected to SDS-PAGE and proteins were transferred onto PVDF membranes (Millipore, Bedford, MA, USA). The membranes were blocked in 130 mM NaCl, 2.5 mM KCl, 10 mM Na_2_HPO_4_, 1.5 mM KH_2_PO_4_, 0.1% Tween-20 and 5% BSA (pH 7.4) for 1 h at room temperature. Then the membranes were probed by primary antibodies overnight at 4 °C. Anti-p-ERK1/2 (MA5–15173) and anti-PCAF (MA5–11186) were purchased from Invitrogen; anti-ERK1/2 (ab17942), anti-H3K9ac (ab4441), anti-H3 (ab12079), anti-HA (ab1424), anti-GFP (ab6556), anti-actin (ab8227), anti-His (ab197049), and anti-MDM2 (ab38618) were all purchased from Abcam (Cambridge, MA). Followed by incubation with the secondary antibody for 1 h at room temperature, the positive signal was detected by using enhanced chemiluminescence (ECL) and analyzed with ImageJ 1.49 (National Institutes of Health, Bethesda, MD, USA).

### Flow cytometric analysis of cell cycle distribution

The transfected SW48 cells in 6-well plates were cultured in serum-deprived medium for 12 h to synchronize cells to G0-phase. Then, the cells were harvested by trypsinisation, washed twice with PBS and fixed in 70% ethanol at 4 °C overnight. The cells were re-suspended in the solution containing 0.2 mg/mL PI (Sigma-Aldrich), 0.1% Triton X-100 (Invitrogen), and 20 μg/mL RNase A (Roche) for 30 min at room temperature in the dark. The percentage of cells in the G0/G1, S and G2/M phases of the cell cycle were analyzed by flow cytometry (FACS Calibur, Becton Dickson, San Jose, CA, USA) and ModFit software (Verity Software House, Topsham, ME, USA).

The article "Ras-ERK1/2 signaling contributes to the development of colorectal cancer via regulating H3K9ac" was retracted in 2021. Reasons: manipulated images; duplicated images; signs of a paper mill; unreliable data.

### Chromatin immunoprecipitation (ChIP)

The transfected SW48 cells (3 × 10^6^ cells per sample) were incubated in 1% formaldehyde for 10 min at room temperature, and the cells were collected and lysed in 200 μL SDS Lysis Buffer (Beyotime). After ultrasonication, the DNA was sheered to an average length of 200–800 bp. The samples were centrifuged at 10,000 *g* at 4 °C for 10 min, and the supernatant was probed by anti-H3K9ac (ab4441, Abcam) and anti-PCAF (MA5–11186, Invitrogen) at 4 °C overnight. The sample treated by anti-IgG (ab190475, Abcam) was used as a blank control. After incubation, 60 μL ProteinA Agarose/SalmonSperm DNA (Thermo Scientific®, Rockford, IL, USA) was added, and the samples were incubated at 4 °C for 2 h. The beads were washed sequentially for 10 min in low-salt wash buffer, high-salt wash buffer, LiCl wash buffer and TE buffer, as previously described [12]. Lastly, the beads were washed in 100 μL 10% SDS, 100 μL 1 M NaHCO_3_, and 800 μL ddH_2_O. 20 μL 5 M NaCl was added, and the crosslinks were reversed for 6 h at 65 °C. RT-qPCR was performed to analyze the amount of immunoprecipitated DNA and input DNA.

### Statistical analysis

Data presented as mean ± SEM. Statistical difference between groups was analyzed by ANOVA following by Duncan post-hoc in SPSS 19.0 software (SPSS Inc., Chicago, IL, USA). A *P*-value of < 0.05 was considered significant.

## Results

### Ras-ERK1/2 repressed H3K9 acetylation in SW48 cells

To examine whether H3K9ac can be modulated by Ras-ERK1/2 pathway, pEGFP-K-Ras^G12V/T35S^ was construct and transfected into SW48 cells. Figure 1a showed that phosphorylation levels of ERK1/2 were remarkably up-regulated in Ras^G12V/T35S^ group as compared to pEGFP group (transfected with an empty plasmid), indicating ERK1/2 pathway was activated by *K-Ras* mutated at G12 V and T35S. Then, the expression changes of H3K9ac were measured by performing Western blot analysis. Results in Fig. 1b and c displayed that, *K-Ras* mutated at G12 V and T35S significantly down-regulated H3K9ac expression (*P* < 0.01), but has no effects on H3 expression. These data suggested that Ras-ERK1/2 activation repressed the acetylation of H3 at lysine 9. In order to reveal whether H3K9 acetylation is specifically mediated by ERK1/2, four inhibitors specific for ERK1/2, MAPK, PI3K and JNK pathways were used, and the expression of H3K9ac was reassessed. As a result, we found that only the inhibitor of ERK1/2 (SCH772984) could recover H3K9ac expression following *K-Ras* mutation at G12 V and T35S (Fig. 1d and e). No such effects were observed in cells treated with the inhibitors specific for MAPK, PI3K and JNK, i.e., SB203580, LY294002 and SP600125. These findings suggested that H3K9 acetylation was specifically mediated by ERK1/2, rather than MAPK, PI3K and JNK.

The article "Ras-ERK1/2 signaling contributes to the development of colorectal cancer via regulating H3K9ac" was retracted in 2021. Reasons: manipulated images; duplicated images; signs of a paper mill; unreliable data.

**Fig. 1:** Ras-ERK1/2 repressed H3K9 acetylation in SW48 cells. SW48 cells were transfected with empty pEGFP vector, pEGFP-K-Ras-WT (wild type) or pEGFP-K-Ras^G12V/T35S^ construct. Protein levels of **a** p-ERK1/2 and **b** and **c** H3K9ac were measured by Western blot analysis. ** *P* < 0.01. Four inhibitors specific for ERK1/2, MAPK, PI3K and JNK pathways, i.e., SCH772984, SB203580, LY294002 and SP600125 were used to treat cells. Protein levels of **d** H3K9ac and **e** p-ERK1/2 were measured by Western blot analysis

### Ras-ERK1/2 repressed H3K9 acetylation to promote the growth and migration of SW48 cells

Next, pEGFP-H3K9Q plasmid was constructed to mimic the acetylated H3K9, and the plasmid was co-transfected with pEGFP-K-Ras^G12V/T35S^ into SW48 cells. Transfection efficiency tested by western blotting revealed that H3K9ac expression was remarkably up-regulated by transfection with pEGFP-H3K9Q, in the presence and absence of pEGFP-K-Ras^G12V/T35S^ (Fig. 2a). MTT assay result showed that, co-transfection of cells with pEGFP-K-Ras^G12V/T35S^ and pEGFP-H3 significantly increased OD-value, compared to the transfection of pEGFP-H3 alone (*P* < 0.001, Fig. 2b). Of note, co-transfection of cells with pEGFP-K-Ras^G12V/T35S^ and pEGFP-H3K9Q attenuated Ras^G12V/T35S^-induced evaluation of OD-value (*P* < 0.001). Same trends were observed in Fig. 2c and d, colony number and OD-value in migration assay were both significantly increased in Ras+H3 group compared to GFP + H3 group (*P* < 0.001). And they were both significantly decreased in Ras+H3K9Q group, as compared to Ras+H3 group (*P* < 0.01). Taken together, recovering the acetylation of H3K9 attenuated the promoting effects of Ras-ERK1/2 on tumor cells growth and migration.

**Fig. 2:** Ras-ERK1/2 repressed H3K9 acetylation to promote the growth and migration of SW48 cells. **a** SW48 cells were transfected with pEGFP-H3, pEGFP-K-Ras^G12V/T35S^ plus pEGFP-H3, or pEGFP-K-Ras^G12V/T35S^ plus pEGFP-H3K9Q (with increasing amount 0.5, 1, and 2 g). **a** Transfection efficiency was tested by Western blot. **b** MTT assay was performed to assess cell viability. Subsequently, pEGFP-H3, pEGFP-K-Ras^G12V/T35S^ plus pEGFP-H3, or pEGFP-K-Ras^G12V/T35S^ plus pEGFP-H3K9Q (2 g) was transfected into cell, and **c** number of colonies and **d** cell migration were respectively determined by colony formation assay and transwell assay. ** *P* < 0.01; *** *P* < 0.001

The article "Ras-ERK1/2 signaling contributes to the development of colorectal cancer via regulating H3K9ac" was retracted in 2021. Reasons: manipulated images; duplicated images; signs of a paper mill; unreliable data.

### Ras-ERK1/2 repressed H3K9 acetylation to affect the transcription of Ras downstream genes

Next, the involvement of H3K9ac in the transcription of Ras downstream genes was addressed. RT-qPCR data in Fig. 3a showed that the mRNA levels of *CYR61* (*P* < 0.01), *IGFBP3* (*P* < 0.01) and *WNT16B* (*P* < 0.05) were significantly up-regulated, while the mRNA levels of *NT5E* (*P* < 0.001), *GDF15* (*P* < 0.01), and *CDC14A* (*P* < 0.01) were significantly down-regulated in Ras+H3 group, as compared to GFP + H3 group. However, the alteration of these mRNAs induced in Ras+H3 group were abolished in Ras+H3K9Q group. ChIP assay results in Fig. 3b showed that H3K9ac level was reduced at the promoters of these genes (*P* < 0.05, *P* < 0.01 or *P* < 0.001) following the activation of Ras-ERK1/2. Based on these data, we speculated that Ras-ERK1/2 mediated the transcription of its downstream genes also via regulating H3K9 acetylation.

**Fig. 3:** Ras-ERK1/2 repressed H3K9 acetylation to affect the transcription of Ras downstream genes. SW48 cells were transfected with pEGFP-H3, pEGFP-K-Ras^G12V/T35S^ plus pEGFP-H3, or pEGFP-K-Ras^G12V/T35S^ plus pEGFP-H3K9Q. **a** RT-qPCR was performed to assess the expression levels of these genes. **b** ChIP was conducted to assess the levels of H3K9ac when different genes were expressed. * *P* < 0.05; ** *P* < 0.01; *** *P* < 0.001

### Silence of HDAC2 recovered H3K9 acetylation and SW48 cells phenotype

Two different sequences of siRNAs specific for *HDAC2* (si-HDAC2–1 and si-HDAC2–2) were transfected into SW48 cells. The mRNA levels of *HDAC2* were remarkably silenced by siRNA transfection (Fig. 4a). Additionally, protein levels of H3K9ac were obviously up-regulated by siRNA transfection, even in K-Ras^G12V/T35S^-expressing cells (Fig. 4b), suggesting H3K9 acetylation could be recovered by HDAC2 silence. Subsequently, cell viability, migration, and cell cycle progression were tested to see the effect of HDAC2 silence on SW48 cells growth and migration. Figure 4c-e demonstrated that both si-HDAC2–1 and si-HDAC2–2 remarkably attenuated the effects of Ras-ERK1/2 activation on SW48 cells viability (*P* < 0.01), migration (*P* < 0.001) and S-phase arrest. And also, the transcription of *CYR61* (*P* < 0.01), *IGFBP3* (*P* < 0.05), *WNT16B* (*P* < 0.05), *NT5E* (*P* < 0.001), *GDF15* (*P* < 0.001), and *CDC14A* (*P* < 0.01) altered by Ras-ERK1/2 activation were attenuated by si-HDAC2–1 plus si-HDAC2–2 (Fig. 4f). These data suggested that silence of *HDAC2* recovered the acetylation of H3K9, which in turn inhibited the growth and migratory capacities of SW48 cells.

The article "Ras-ERK1/2 signaling contributes to the development of colorectal cancer via regulating H3K9ac" was retracted in 2021. Reasons: manipulated images; duplicated images; signs of a paper mill; unreliable data.

**Fig. 4:** Silence of HDAC2 recovered H3K9 acetylation and SW48 cells phenotype. **a** The efficiency of siRNA-mediated HDAC2 silence was determined. **b** SW40 cells were transfected as indicated. The expression changes of H3K9ac were detected by Western blot analysis. **c** Cell viability, **d** migration, **e** cell cycle progression, and **f** several gene transcription were respectively assessed by MTT assay, transwell assay, flow cytometry and RT-qPCR. * *P* < 0.05; ** *P* < 0.01; *** *P* < 0.001

### Ras-ERK1/2 repressed H3K9 acetylation in SW48 cells via degradation of PCAF

In order to reveal how Ras-ERK1/2 repressed H3K9 acetylation, we focused on investigating *PCAF*, a reported upstream gene of H3K9ac [13]. Figure 5a displayed that mRNA levels of *PCAF* and *HDAC2* were both unaffected by K-Ras^G12V/T35S^. Figure 5b results indicated that the protein level of PCAF was down-regulated by K-Ras^G12V/T35S^, but the protein level of HDAC2 was unaffected. These results implied that Ras-ERK1/2 post-transcriptionally down-regulated PCAF expression. This was also confirmed in Fig. 5c, that both PCAF and H3K9ac protein expression was repressed in Ras^G12V/T35S^ group. To further confirmed whether PCAF involved in the transcription of Ras downstream genes, ChIP was performed. Results from Fig. 5d showed that all of these genes that exhibited reduced H3K9ac following Ras-ERK1/2 activation also exhibited significant reduction in PCAF binding, suggesting PCAF was responsible for Ras-ERK1/2-repressed H3K9 acetylation.

**Fig. 5:** Ras-ERK1/2 repressed H3K9 acetylation in SW48 cells via degradation of PCAF. **a** The mRNA level of PCAF after the indicated transfected was tested. **b** and **c** Western blot analysis was performed to measure the expression of PCAF, HDAC2, and H3K9ac following the indicated transfection. Anti-HA antibody was used for testing the exogenous levels of PCAF and HDAC2. **d** ChIP analysis for testing PCAF levels when different genes were expressed. **e** 25 μM of MG132 was used to treat cells, after which Western blot was performed to reassess PCAF level. Protein expression of H3K9ac was monitored in the **f** absence or **g** presence of MG132. ** *P* < 0.01; *** *P* < 0.001

Finally, SW48 cells were treated with MG132 (a proteasome inhibitor) to confirm whether PCAF regulated H3K9ac post-transcriptionally. Figure 5e showed that MG132 remarkably reversed the reduction of PCAF in K-Ras^G12V/T35S^-expressing cells. Results in Fig. 5f showed that H3K9ac levels were down-regulated by Ras^G12V/T35S^ after 48 h of transfection in absence of MG132. However, treating cells with 25 μM MG132 gradually recovered the expression of H3K9ac (Fig. 5g). Thus, it is possible that Ras-ERK1/2 pathway repressed H3K9 acetylation through regulating PCAF.

The article "Ras-ERK1/2 signaling contributes to the development of colorectal cancer via regulating H3K9ac" was retracted in 2021. Reasons: manipulated images; duplicated images; signs of a paper mill; unreliable data.

### Ras-ERK1/2 regulated H3K9ac via MDM2-mediated PCAF degradation

It has been reported that the E3 ubiquitin ligase MDM2 could bind to acetylases, such as p300/CBP or PCAF [14]. Thus, we explored whether MDM2 was implicated in PCAF degradation in K-Ras^G12V/T35S^-expressing cells. Figure 6a and b showed that PCAF expression was gradually repressed with MDM2 expression. However, in MDM2-mutant (MDM2-MU) transfected cells, no such down-regulations were observed in PCAF expression (Fig. 6c and d), indicating MDM2 was responsible for PCAF degradation.

**Fig. 6:** Ras-ERK1/2 regulated H3K9ac via MDM2-mediated PCAF degradation. SW48 cells were transfected with pEGFP-K-Ras^G12V/T35S^, PCAF-HA, MDM2-His (with increasing amount 0.5, 1, and 2 g) and pEGFP-N1. **a** Exogenous and **b** endogenous expression of PCAF was measured by Western blot. SW48 cells were transfected either by MDM2-His (2 g) or by MDM2 mutated type (MDM2-MU), then **c** exogenous and **d** endogenous expression of PCAF were reassessed. Anti-His and anti-HA antibodies were used for testing the exogenous levels of MDM2 and PCAF, respectively. **e** MDM2 and H3K9ac expression in cells transfected with pEGFP-K-Ras^G12V/T35S^ or pEGFP-N1. **f** The protein level of MDM2 after siRNA transfection was tested. **g** After the indicated transfection, H3K9ac level was tested by Western blot

Next, we established a link between H3K9ac expression and MDM2 activity to reveal whether MDM2-mediated PCAF degradation was required to modulate Ras-ERK1/2-repressed H3K9 acetylation. Figure 6e showed that, MDM2 was up-regulated, while H3K9ac was down-regulated in K-Ras^G12V/T35S^-expressing cells. Thereafter, the expression of MDM2 was repressed in K-Ras^G12V/T35S^-expressing cells by siRNA transfection (Fig. 6f). As a result, we found that silence of MDM2 resulted in an up-regulation of H3K9ac in K-Ras^G12V/T35S^-expressing cells (Fig. 6g). Collectively, these data implied that Ras-ERK1/2 regulates H3K9ac via MDM2-mediated PCAF degradation.

## Discussion

In physiological conditions, inactive Ras (GDP-bound) switches to active form (GTP-bound), and activates MEK kinase, which in turn activates ERK kinase. The activation of ERK subsequently phosphorylates a number of substrates, and thereby modulates cell fate [15]. Although *Ras* acted as a control switch in the activation of many signaling pathways, it seems that ERK is one of the most important pathways which can be activated by *Ras* point mutation [16]. This was also confirmed in this study, that *K-Ras* mutated at G12 V and T35S induced a significant activation of ERK1/2 signaling. Since hyperactivation of Ras-ERK signaling pathway appears frequently in cancers, this signaling has been considered as a promising target for controlling of cancers [15]. However, the molecular regulation following by Ras-ERK activation is still unclear. This work demonstrated that activation of Ras-ERK could significantly repress the acetylation of H3K9 through MDM2-dependent PCAF degradation. And also, the repressed H3K9ac contributed to colorectal cancer SW48 cells growth, migration, and the transcription of several tumor-associated genes.

The article "Ras-ERK1/2 signaling contributes to the development of colorectal cancer via regulating H3K9ac" was retracted in 2021. Reasons: manipulated images; duplicated images; signs of a paper mill; unreliable data.

Histone H3 acetylation is a well-known modification process, which is often marks for the open up of chromatin and activation of gene transcription [17]. To date, five isoforms of acetylated histone H3 proteins have been found. Depending on the acetylation sites of histone H3, they are named as histone H3 acetylation at lysine 9 (H3K9ac), 14 (H3K14ac), 18 (H3K18ac), 23 (H3K23ac) and 27 (H3K27ac). The acetylation of histone H3 has clinical diagnostic significance in many cancers, including epithelial ovarian tumor [18], hepatocellular carcinoma [19], oral cancer [8], and cervical cancer [20]. Among these acetylated histone H3, H3K9ac is the most widely studied one in cancer and other diseases. It has been suggested that H3K9 acetylation can be triggered by external stimuli, such as long-term alcohol consumption [21], and traffic-related air pollution [22]. Our study for the first time suggested that H3K9 acetylation can be specifically catalyzed by Ras-ERK1/2 signaling, rather than MAPK, PI3K and JNK signaling.

The role of H3K9ac in colorectal cancer has been sporadically studied. Lutz et al., demonstrated that high levels of H3K9ac were frequently occurred in patients with colorectal cancer [23]. Another study demonstrated that the expression pattern of H3K9ac was altered during aging, which is a prime risk factor of the development of colorectal cancer [24]. These two studies suggested H3K9ac as a potential target for novel treatment option of colorectal cancer. However, a contrary finding was reported by Nakazawa et al., who demonstrated that H3K9ac expression was unchanged between normal and neoplastic cell nulei in the colorectal cancers [25]. Based on these previous studies, the role of H3K9ac in colorectal cancer is confusing. Herein, we attempted to study the in vitro effects of H3K9ac on colorectal cancer cells growth and migration, in order to reveal the exact function of H3K9ac in this cancer. By using a mimicked H3K9ac expression vector (H3K9Q), the expression of H3K9ac in K-Ras^G12V/T35S^-transfected SW48 cells was recovered. As a result, the growth and migratory capacities of SW48 cells were both reduced, suggesting the acetylation of H3K9 contributed to colorectal cancer SW48 cells growth and migration following Ras-ERK1/2 activation.

The article "Ras-ERK1/2 signaling contributes to the development of colorectal cancer via regulating H3K9ac" was retracted in 2021. Reasons: manipulated images; duplicated images; signs of a paper mill; unreliable data.

There are several genes have been found to be transcriptionally regulated by H3K9ac following Ras-ERK1/2 activation in this study, further suggested H3K9ac as a downstream effector of Ras-ERK1/2 signaling. All of the studied genes are known to be closely related with tumor cells growth and migration. *CYR61* expression was associated with poor prognosis in patients with colorectal cancer [26] and it promotes cancer cells proliferation, invasion, survival, and metastasis [27, 28]. In addition to *CYR61*, *IGFBP3* [29] and *GDF15* [30] are also effective predictors of outcomes in patients with colorectal cancer. *WNT16B* [31], *NT5E* [32], *GPF15* [33], and *CDC14A* [34] are implicated in tumorigenesis via regulating tumor growth and EMT process. According to the findings reported elsewhere, *CYR61* [35], *NT5E* [36], *WNT16B* [37] and *GDF15* [38] were identified as oncogenes, while *IGFBP3* [39] and *CDC14A* were found to be tumor-suppressive genes. In the current study, the expression of *CYR61*, *IGFBP3*, *WNT16B* was found to be down-regulated, whereas the expression of *NT5E*, *GDF15*, *CDC14A* was found to be up-regulated by H3K9ac. This phenomenon indicates the impacts of H3K9ac on colorectal cancer cells are complex, since both oncogenes and tumor-suppressive genes can be up-regulated or down-regulated by H3K9ac. Additional investigations are required to further analyze the pleiotropic effects of H3K9ac on cancer.

HATs and HDACs are two kind of key enzymes in catalyzing the acetylation and deacetylation of H3. Human HDACs can be divided into several large families: HDAC I (HDAC1, 2, 3 and 8), HDAC II (HDAC4, 5, 6, 7, 9 and 10), HDAC III (Sirt1-Sirt7), and HDAC IV (HDAC11) [40]. Human HATs include TIP60, MOZ/MYST3, MORF/MYST4, HBO1/MYST2, MOF/MYST1, P300, CBP, GCN5, PCAF, and ELP3 [41]. HDAC2 is highly expressed in patients with early stages of colorectal cancer, and the elevated HDAC2 expression is associated with the poor prognosis [42, 43]. In this study, we confirmed H3K9ac can be deacetylated by HDAC2 by using siRNAs specific for HDAC2. Besides, it seems that silence of HDAC2 recovered H3K9ac expression and SW48 cells phenotype following Ras-ERK1/2 activation. And also, we indicated that H3K9 was acetylated by PCAF. Moreover, the acetylation of H3K9 by PCAF was through a MDM2-dependent fashion.

The article "Ras-ERK1/2 signaling contributes to the development of colorectal cancer via regulating H3K9ac" was retracted in 2021. Reasons: manipulated images; duplicated images; signs of a paper mill; unreliable data.

## Conclusions

In conclusion, this study demonstrated that H3K9ac was a specific target for Ras-ERK1/2 signaling pathway. H3K9 acetylation can be modulated by HDAC2 and MDM2-depedent degradation of PCAF. The revealed regulation provides a better understanding of Ras-ERK1/2 signaling in tumorigenesis and the findings will accelerate the development of novel targets for colorectal cancer treatment.
